# The Ensemble Machine Learning-Based Classification of Motor Imagery Tasks in Brain-Computer Interface

**DOI:** 10.1155/2021/1970769

**Published:** 2021-11-09

**Authors:** Abdulhamit Subasi, Saeed Mian Qaisar

**Affiliations:** ^1^Institute of Biomedicine, Faculty of Medicine, University of Turku, Kiinanmyllynkatu 10, Turku 20520, Finland; ^2^College of Engineering, Effat University, Jeddah 22332, Saudi Arabia; ^3^Communication and Signal Processing Lab, Energy and Technology Research Center, Effat University, Jeddah 22332, Saudi Arabia

## Abstract

The Brain-Computer Interface (BCI) permits persons with impairments to interact with the real world without using the neuromuscular pathways. BCIs are based on artificial intelligence piloted systems. They collect brain activity patterns linked to the mental process and transform them into commands for actuators. The potential application of BCI systems is in the rehabilitation centres. In this context, a novel method is devised for automated identification of the Motor Imagery (MI) tasks. The contribution is an effective hybridization of the Multiscale Principal Component Analysis (MSPCA), Wavelet Packet Decomposition (WPD), statistical features extraction from subbands, and ensemble learning-based classifiers for categorization of the MI tasks. The intended electroencephalogram (EEG) signals are segmented and denoised. The denoising is achieved with a Daubechies algorithm-based wavelet transform (WT) incorporated in the MSPCA. The WT with the 5th level of decomposition is used. Onward, the Wavelet Packet Decomposition (WPD), with the 4th level of decomposition, is used for subbands formation. The statistical features are selected from each subband, namely, mean absolute value, average power, standard deviation, skewness, and kurtosis. Also, ratios of absolute mean values of adjacent subbands are computed and concatenated with other extracted features. Finally, the ensemble machine learning approach is used for the classification of MI tasks. The usefulness is evaluated by using the BCI competition III, MI dataset IVa. Results revealed that the suggested ensemble learning approach yields the highest classification accuracies of 98.69% and 94.83%, respectively, for the cases of subject-dependent and subject-independent problems.

## 1. Introduction

A Brain-Computer Interface (BCI) allows individuals to use electroencephalogram (EEG) signals to operate external equipment such as virtual worlds, robots, or spelling machines. The fundamental objective of the BCI is to use brain signals to create the required commands to control peripherals. The most important application is to bypass injured areas of the body or stimulate partly paralyzed organs. BCI devices are viewed as the best solution to mitigate problems for persons with various neuromuscular impairments such as spinal cord damage, amyotrophic lateral sclerosis, cerebral palsy, and stroke [1].

BCI systems may be divided into two categories based on the EEG signals collection methods: noninvasive and invasive. Because of the ease of usage, much current research has focused on noninvasive BCIs. Event-related potentials, steady-state visual-evoked potentials, and slow cortical potentials are the three main noninvasive BCI approaches [2]. In noninvasive approach, different EEG signals can be utilized in BCI. Within the EEG alpha and beta frequency regions of the brain signals, BCI systems typically employ Motor Imagery approaches to produce event-related actions. This form of BCI is mostly utilized for cursor control on computer screens and wheelchair navigation or in virtual environments. Several Motor Imagery (MI) techniques are commonly used, including tongue movement, left/right hand movement, foot movement, and mental counting [3]. The goal of BCI technology is to assist people with brain diseases including cerebral palsy, amyotrophic lateral sclerosis, and motor neuron disease. EEG is commonly used as a tool for the BCI system [4, 5]. Based on phenomena of event-related synchronization (ERS) and event-related desynchronization (ERD), scientists can interpret and identify MI-related brain signals. The translation of imagination to action involves ERS and ERD. Both ERD and ERS are presented by variations in the EEG signal's oscillatory behaviour and can be investigated by the time-frequency analysis to identify the MI tasks [6]. MI is characterized as a human brain's ability to resynthesize motor experiences with no obvious movement. Such mental images may both appear consciously and be created and controlled deliberately by a subject making MI, which is a flexible and usable method for examining processes of human cognition and motor activity. As various studies have shown, MI uses almost the same neural framework as motor execution, which enables motor activity to be altered by MI training. The MI-based BCI uses variations in the cortical sensorimotor rhythms (SMR), generally ERD related to the different sensorimotor events, including MI [7]. In addition, BCI may serve as a technical bridge for the management of Active and Assisted Living (AAL) systems in the sense of intelligent environments and smart homes. As with any other traditional AAL device interface, the consumer needs to view BCI-enabled control as simple and normal as possible in order to encourage BCI acceptance and effectiveness [8].

Computer-based automated MI signal detection is essential for providing continuous assistance to the intended patients. The preprocessing, feature extraction, dimension reduction, and classification are all parts of the EEG-based automated MI signal detection approaches [9, 10].

Feature extraction and dimension reduction are the most critical aspects of the classification system for EEG-based MI signals since they greatly affect classifier efficiency and computational complexity. If the features retrieved from EEG signals include irrelevant characteristics, the classifier's performance will suffer. The amount of features determines the classifier's processing cost. As a result, extracting the appropriate amount of relevant features from EEG-based MI signals is critical for achieving high classification performance and computational effectiveness for a classifier [9]. In this study, the dataset IVa from the BCI competition is utilized in the experiments [11]. AA, AL, AV, AW, and AY are codes of five healthy participants that contributed to this dataset. Two classes of MI activities, right hand and right foot movement, referred to as class 1 and class 2, respectively, are involved.

### 1.1. Contribution

The main objective of this work is to extract relevant features from the EEG signals and to design a classifier that can effectively recognize the intended MI tasks.

The major contributions are to propose a novel hybridization of the Multiscale Principal Component Analysis (MSPCA), Wavelet Packet Decomposition (WPD), subbands statistical features selection, and ensemble learning technique for automated classification of the MI tasks. The functional steps are as follows:

- The Multiscale Principal Component Analysis (MSPCA) is used for denoising.
- The Wavelet Packet Decomposition is used for producing the subbands.
- The six different statistical features are extracted from each subband. These are mean absolute value, power, standard deviation, skewness, kurtosis, and ratio of absolute mean values of adjacent subbands.
- The extracted features are passed to the proposed ensemble learning-based classifiers for automated identification of the MI tasks.

### 1.2. Organization

The remainder of the paper is organized as follows.  Section 2 presents a literature review. In Section 3, materials and methods are introduced, Section 4 discusses the results, and the conclusion is presented in Section 5.

## 2. Literature Review

The loss of motor function is one of the most concerning effects of injury or disease to the nervous system. The BCI assistive technologies have allowed artificial prostheses, wheelchairs, and computers to be controlled by the electrical activity of the brain in this decade. The major challenges in the BCI systems are precision and processing effectiveness. The current systems have high computational complexity and need advanced and resourceful processing systems to attain a real-time response. Additionally, their classification performance and robustness need to be improved. In this context, several studies have been presented [12, 13].

Zarei et al. [9] used a combination of the Principal Component Analysis (PCA) and the cross-covariance (CCOV) method for features extraction from the EEG signals for the BCI application. The multilayer perceptron neural networks (MLP) and Least Square Support Vector Machine (LS-SVM) are used for classification. The performance of the system is tested by using the BCI competitions dataset IVa. Kayikcioglu and Aydemir [10] extracted features from the EEG signals by using two-dimensional features mining from the 2nd order polynomial coefficients. Then, the functions are categorized using the algorithm k-nearest neighbor (k-NN). They achieved considerable enhancement in speed and accuracy while evolving the performance for the dataset Ia from the 2003 BCI competition. Leamy et al. [12] conducted a comparative experimental research, from a machine learning perspective, for MI-related EEG features in stroke subjects. They try to explore if such features are generalizable to use trained machine learning parameters employing healthy subjects and stroke-affected patients. If BCI is trained with appropriate data, it gives relatively good results to stroke patients; then such a deployment model will make BCI far more realistic in a clinical setting for stroke recovery. On the other hand, if the stroke-affected EEG is significantly different from healthy EEG or changes over time, it may need more sophisticated architecture from a machine learning perspective for the realistic implementation of BCI in such a setting.

Li et al. [13] proposed a new approach for MI pattern identification. It combines a common spatial pattern algorithm for frequency band selection and features selection, and the classification is carried out with the particle swarm optimized twin Support Vector Machine. They used datasets IIb of BCI competition IV to test the proposed system. For a classification task, Kevric and Subasi [14] employed MSPCA-based denoising of the EEG signals. Comparison among three features extraction techniques, namely, the Empirical Mode Decomposition (EMD), Discrete Wavelet Transform (DWT), and WPD, is conducted. The extracted features sets are classified by using the k-Nearest Neighbor (k-NN) algorithm. The system performance is tested by using the publicly available BCI competition III dataset IVa. Miao et al. [15] have suggested an EEG signals channel selection method. It uses the linear discriminant criteria for automated selection of channels with strong discriminative capabilities. Furthermore, the artificial bee colony algorithm is used for dimension reduction. The performance is tested by using the dataset IVa from the BCI competition III. In [16], Baali et al. have used a signal-dependent orthogonal transformation for features extraction. The classification is carried out by using a tree-based logistic model classifier. In [17], Chaudhary et al. used the flexible analytic wavelet transform (FAWT) for features extraction. The classification is carried out with ensemble learning-based subspace k-Nearest Neighbor (k-NN) classifier. In [18], Rahman et al. have used the Rényi min-entropy-based features extraction approach. The extracted features are used for classifying 4 different BCI categories by using the Random Forest (RF) algorithm. The performance of the proposed method is evaluated by using the BCI competition IV dataset.

Khare and Bajaj [19] employed the extreme learning machine-based classification of the MI tasks. The channels selection is realized by using the multicluster unsupervised learning approach. The signal decomposition is performed by using a flexible variational mode decomposition (F-VMD). Pertinent features from different modes are explored, namely, hjorth, entropy, and quartiles. In [20], the authors have used the flexible analytic wavelet transform (FAWT) for signal decomposition. Time-frequency attributes are calculated from subbands. The PCA, kernel PCA (KPCA), locally linear embedding (LLE), and Laplacian Eigenmaps (LE) are used for feature selection. The Linear Discriminant Analysis (LDA) algorithm is used for the classification. The performance is tested by using the BCI competition III dataset IIIb.

Tiwari et al. [21] proposed a Deep Neural Network (DNN) model for automated identification of the MI tasks by utilizing the EEG signals. The Power Spectral Densities (PSDs) are extracted as features from subbands by applying a bank of Butterworth filters. The performance is tested for the BCI competition III and V dataset MI tasks. Musallam et al. [22] utilized a Convolutional Neural Network (CNN) model that incorporates a number of different methods, including temporal convolutional networks (TCNs), separable convolution, depthwise convolution, and layer fusion. The intended EEG signals are processed by two successive 1D convolution stages. The first in the time domain and subsequently channelwise and the second based on the image-like representation are used as an input of the main TCN. The performance is tested by using the BCI competition IV, IIa dataset.

## 3. Materials and Methods

The proposed system's framework is shown in Figure 1. A description and parameterization of different system modules are given in the following section.

### 3.1. Dataset

The suggested system performance is evaluated by using the well-known BCI competition III, dataset IVa^1^ [11]. **AA**, **AL**, **AV**, **AW**, and **AY** are codes of five healthy participants that contributed to this dataset. They completed two classes of MI activities involving right hand and right foot movement, referred to as class 1 and class 2, respectively. Subjects are seated in comfortable chairs with armrests. The EEG signals are acquired from 118 electrodes, mounted by following the 10/20 globally accepted standard. Each considered subject performed 140 trials of each category. Being two considered classes of tasks, it resulted in a total of 280 trials per subject. Each trial is carried out for a duration of 3.5 sec. For each category, the data is made up of different-sized training and testing sets.

The training set for subjects **AA**, **AL**, **AV**, **AW**, and **AY** has 168, 224, 84, 56, and 28 trials, respectively. The testing set consists of 112, 56, 196, 224, and 252 trials for participants **AA**, **AL**, **AV**, **AW**, and **AY**, respectively.

The EEG signals are originally recorded at a rate of 1 kHz. These EEG signals are bandlimited to 50 Hz by using digital filtering and are onward downsampled to the rate of 100 Hz [11]. These downsampled versions of signals are used in this study. The EEG signals from only three channels (C3, Cz, and C4) are selected from a total of 118 available channels. This is because these channels contain the most discriminatory features on Motor Imagery activities involving the hands and feet. For each patient, 280 EEG segments of 3.5 seconds, with 3 selected channels, are prepared [11]. These are from two categories: right hand and foot. In total, 1400 EEG instances were used for the five mentioned subjects. They belong to the two considered classes of the MI tasks.

### 3.2. Denoising with Multiscale Principal Component Analysis (MSPCA)

In multivariate statistical analysis, the PCA is one of the most important models. Let a measurement dataset with *m* sensors exist, such as *xϵR*^*m*^. Each sensor in the measurement sample contains *n* separate sampling data, which are combined into a data matrix of size *mxn*. The process is given by

(1) $$\begin{array}{c} X=\left[x_{1},\;x_{2},\;x_{3},\ldots ,x_{n}\right]. \end{array}$$

Each row of *X* represents a sample, and each column represents a measurement variable. The PCA model begins by standardizing each sample of *X* by computing the covariance matrix of *X*. The process is given by

(2) $$\begin{array}{c} \text{cov}\left(x\right)\approx \frac{X^{T}.\;X}{n-1}. \end{array}$$

The size of the feature values is ordered from large to small when the feature decomposition of *X* is done. The process of decomposing *X* in its principal components is given by equation (3), where *PϵR*^*m*×*A*^ contains first *A* feature vectors of cov(*x*). *TϵR*^*n*×*A*^ is a matrix, where each column is known as the principal element variable. *A* is the count of principal components, and it is equal to the number of columns in *T*.

(3) $$\begin{array}{c} \left\{\begin{array}{c} X=\hat{X}+Er=T.P^{T}+Er,\\ T=X.P. \end{array}\right. \end{array}$$

Equation (4) can be used to determine the principal component's covariance, where *λ*_1_,  *λ*_2_,   …,  *λ*_*n*_ are the first *A* large eigenvalues of the covariance matrix of *X*.

(4) $$\begin{array}{c} \Lambda =\frac{X^{T}.X}{n-1}=\left[\begin{array}{c} \lambda_{1}\ldots \ldots \cdot \cdot \\ \ldots \cdot \lambda_{2}\ldots \cdot \\ .\\ .\\ \ldots \ldots \ldots \cdot \lambda_{n} \end{array}\right]. \end{array}$$

In this paper, the wavelet transform is combined with the Principal Component Analysis (PCA) to create MSPCA for the incoming signal denoising purpose. The principle of wavelet transform is described in Section 3.3. In this study, the 5th level of decomposition is realized by using the Daubechies wavelet analysis algorithm [23]. MATLAB is used for implementing the wavelet transform [24].

The ability of standard PCA is enhanced by incorporating the multiscale analysis. Collectively, it results in the multiscale PCA (MSPCA) [25]. In MSPCA, the PCA's capacity to extract covariance between variables is combined with orthonormal wavelets' ability to distinguish deterministic features from stochastic processes and approximately decorrelate the autocorrelation across observations. It identifies linearly related wavelet coefficients at multiple level subbands, obtained with wavelet transform. It allows representing each considered subband with fewer features while removing the autocorrelated coefficients. It results in a simplified representation of the considered subbands at each level of decomposition. The EEG waveforms are decomposed by using the Daubechies wavelet analysis algorithm with the 5th level of decomposition. In the next step, the PCA of detailed coefficients, obtained at each level, is utilized to select the principal components at each scale. Onward, the signal is reconstructed by using the wavelet synthesis. It diminishes the unwanted noise from the incoming signal and generates a simple and noise-free signal version [25, 26]. MATLAB is used for implementing the MSPCA [24].

### 3.3. Features Extraction with Wavelet Packet Decomposition (WPD)

Wavelets are well-known functions and widely used for multiresolution time-frequency analysis. Wavelets can be mathematically described by equation (5) [23], where the dilation parameter is represented by *s* and the translation parameter is represented by *u*. The parameters can be generated at the same time with different frequencies.

(5) $$\begin{array}{c} \psi \left(t\right)=\frac{1}{\sqrt{S}}\psi \left(\frac{\left(t-u\right)}{s}\right). \end{array}$$

The process of decomposing a signal *x* (*t*), by using wavelet transform, can be given by

(6) $$\begin{array}{c} W_{X}\left(u,s\right)=\frac{1}{\sqrt{S}}\int_{-\infty }^{+\infty }x\left(t\right)\psi^{*}\left(\frac{\left(t-u\right)}{s}\right)\text{d}t. \end{array}$$

A discrete version of the wavelet transform (DWT) is used in this study. The selection of the right number of wavelet decomposition levels, *m*, is the first key step in the DWT decomposition. The incoming signal *x*[*n*] passes concurrently through both the high-pass and low-pass filters, *h*[*k*] and *l*[*k*]. For the *m*^*th*^ scale level, the output is represented by two subbands, namely, Detail (*D*_*m*_) and Approximation (*A*_*m*_). The process is clear from equations (7) and (8), where *H* is the order of filters used at different decomposition stages:

(7) $$\begin{array}{c} D_{m}\left[k\right]\sum_{k=1}^{H}x\left[n\right].h\left[2.k-n\right], \end{array}$$

(8) $$\begin{array}{c} A_{m}\left[k\right]\sum_{k=1}^{H}x\left[n\right].l\left[2.k-n\right]. \end{array}$$

The Wavelet Packet Decomposition is known as the extension of Discrete Wavelet Transform (DWT). The DWT mainly focuses on the low-frequency components, known as approximate coefficients. However, WPD utilizes both approximate and detailed coefficients, high-frequency components [27]. Consequently, when tactfully used, the WPD can result in signal decomposition with superior frequency resolution compared to the DWT [26]. In the studied case, the denoised signal is further analysed by using four levels of WPD. Pertinent statistical features are extracted from multiresolution subbands, obtained with the 4th level of WPD. MATLAB is used for implementing the WPD [24]. The principle of employed WPD with the 4th level of decomposition is shown in Figure 2, where *D*_*m*_ and *A*_*m*_ are, respectively, detailed and approximation coefficients at different decomposition stages and *mϵ*{1,  2,  3,  4}.

### 3.4. Dimension Reduction

Since the dimension of the extracted features with WPD is high, the dimension should be reduced. Therefore, in this study, the dimension of extracted features is reduced by using statistical values of the WPD subbands. Using the statistical values of the subbands, the pertinent classifiable features are created from 16 subbands, shown in Figure 2. Five features are extracted from each subband, namely, mean absolute value, average power, standard deviation, skewness, and kurtosis. It results in 16 × 5=80 features. Additionally, the ratios of absolute mean values of the adjacent subbands are computed, resulting in 15 more features. In this way, in total, 95 features are extracted for each EEG instance, resulting in feature set dimension of 1400 × 95 for all considered instances.

### 3.5. Classification Methods

The prepared features set is categorized by using k-Nearest Neighbor (k-NN), C4.5 Decision Tree, REP Tree, Support Vector Machine (SVM), Random Tree (RT), and RF, which are all well-known robust classification algorithms. Weka is used for evaluating the considered classifiers [28, 29]. To avoid any bias in findings due to the limited volume of the dataset, the 10-fold cross-validation (10-CV) approach is used along with multiple evaluation measures, namely, accuracy, F-measure, and the area under the ROC curve (AUC). Here, ROC stands for receiver operating characteristic [29].

#### 3.5.1. Support Vector Machine (SVM)

The SVM searches for hyperplane in an N-dimensional space in the classification of the data points. The SVM can be used for both classification and regression. The system functions by focusing on the decision line. It is a theoretically mature algorithm, only takes tens of instances for training, and is unaffected by the number of dimensions. Furthermore, effective approaches are developed to rapidly train this classifier [30]. In this study, the SVM is used with the cubic polynomial kernel and with a regularization parameter of 100.

#### 3.5.2. K-Nearest Neighbor (k-NN)

The k-NN refers to a supervised learning algorithm used in regression and classification problems. The algorithm functions by assuming that every data falling near each other belongs to the same class. It means that the algorithm considers that the classification of information is based on similarities. The technique is highly preferred because of its simplicity [30]. In this study, the k-NN with *k*=1 is used. Here, *k* is the number of neighbors, used in the decision.

#### 3.5.3. REP Tree

REP Tree creates a decision or regression tree using information variance reduction and then prunes it using reduced-error pruning. It optimizes speed by only sorting values for numeric attributes once. The minimum number of instances per leaf, maximum tree depth, minimum fraction of training set variance for a split, and the number of folds for pruning are adjustable parameters [31]. In this study, the REP Tree is used with its default configurations, available in Weka [28, 29].

#### 3.5.4. C4.5 Decision Tree

The C4.5 can create classifiers that are redescribed as rulesets. C4.5 starts by growing an initial tree using the divide-and-conquer method. It labels the potential test instances by using two heuristic criteria. The first is the information gain, which tries to minimize the total entropy of subsets. The second is the default gain ratio, which tries to divide the information gain by the information supplied via the test outcomes [30]. In this study, the C4.5 is used with its default configurations, available in Weka [28, 29].

#### 3.5.5. Random Tree (RT) Classifiers

The RT is a supervised learning algorithm that is easy to use and flexible. The algorithm produces excellent results despite lacking hyperparameter tuning. A combination of decision subtrees is trained based on the bagging method. The primary concept of the functioning of the Random Tree is that combined learning models will increase the quality of results gained [31]. In this study, the RT is used with its default configurations, available in Weka [28, 29].

#### 3.5.6. Random Forests (RF)

The RF refers to a robust machine learning algorithm for various tasks such as classification and regression. The algorithm works by using bagging and randomness when creating each of the trees. It makes an uncorrelated forest of trees where their prediction is more accurate than a single tree [32]. In this study, the RF is used with 100 trees.

#### 3.5.7. Rotation Forest (RoF)

The RoF is a feature extraction-based classifier ensemble. We make the training data for a basic classifier by randomly partitioning the feature set into *Q* subgroups. PCA is applied to each subgroup, and *Q* is a parameter of the method. To retain the data's variability information, all basic components are kept. As a result, rotating the *Q*-axis produces additional attributes for a base classifier [33]. All primary components are kept in order to preserve the data's variability information. As a result, new features for a base classifier are formed by rotating the *Q*-axis [33]. The purpose of the rotation approach is to enhance individual accuracy while also providing variation within the group. Each base classifier's feature extraction contributes to diversity.

#### 3.5.8. The Random Subspace Method (RSM)

A well-known ensemble technique is the RSM [34]. The training data is also modified in the RSM. This change, however, is done in the feature space. The *B*-dimensional random subspace of the original *B*-dimensional feature space is thus obtained. As a result, the updated training set has *B*-dimensional training objects in it. Then, in the final decision rule, classifiers can be built in random subspaces and combined using simple majority voting [35].

### 3.6. The Ensemble Learning Method

The ensemble learning methods can improve the performance of classification [26]. In this framework, the RoF and the RSM classifiers are employed with single classifiers. Multiple classifiers are used for the considered classification task. Findings of classifiers with various accuracies are combined via an ensemble-based approach [36]. The principle is depicted with the help of Figure 3.

For the case of RoF, by randomly splitting the features set into *Q* subgroups, we generate training data for a base classifier. After that, the PCA is applied to each subgroup. To maintain the data's variability information, all principal components are taken into consideration. This is how *Q*-axis rotations are realized to prepare new features for a base classifier. The rotation technique is designed to enhance individual accuracy while simultaneously fostering variation within the ensemble. Each base classifier's diversity is created by feature extraction. In this scenario, accuracy is measured by training each base classifier with the entire dataset [33].

For the case of RSM, the *B*-dimensional random subspace of the original features set was produced. As a result, the training set comprises *B*-dimensional training objects. In this approach, we built classifiers in random subspaces and used simple majority voting to aggregate their results [35].

### 3.7. Performance Evaluation Measures

In order to avoid any bias in the classification performance evaluation, multiple evaluation measures, namely, accuracy, F-measure, and AUC, are utilized [29]. The accuracy is defined by equation (9). True positives, true negatives, false positives, and false negatives are represented as tp, tn, fp, and fn, respectively. The F-measure is given by equation (10). The AUC presents the classification performance graphically. It is the area under the curve of the graph, obtained by tracing the True Positive Rate (TPR) with respect to the False Positive Rate (FPR). The TPR and FPR are, respectively, given by equations (11) and (12).

(9) $$\begin{array}{c} \text{accuracy}\left(\text{ACC}\right)=\frac{tp+tn}{tp+tn+fp+fn}\times 100\text{ ,} \end{array}$$

(10) $$\begin{array}{c} F-\text{measure}=\frac{tp}{tp+1/2\left(fp+fn\right)}, \end{array}$$

(11) $$\begin{array}{c} \text{TPR}=\frac{tp}{\left(tp+fn\right)}, \end{array}$$

(12) $$\begin{array}{c} \text{FPR}=\frac{fp}{\left(fp+tn\right)}. \end{array}$$

## 4. Results

The system performance is tested by using the BCI competition III, dataset IVa [11]. An example of the input EEG signal and its denoised version, obtained with the MSPCA, is shown in Figure 4.

The denoised signal is onward decomposed in 16 subbands by using the 4th level of WPD. An example of obtained subbands is shown in Figure 5.

The overall system performance is studied in terms of classification precision. Findings are outlined in Table 1. These results are also presented graphically. In Figure 6, the accuracy scores, obtained with different classifiers, are shown. Figures 7 and 8, respectively, show the F-Measure and AUC values, obtained with different classifiers.

It is evident from Table 1 that the ensemble of k-NN and RoF attains the superior classification performance in most of the cases, compared to the other studied classifiers. The obtained percentages accuracies obtained for subjects **AA**, **AL**, **AV**, **AW**, and **AY** are, respectively, 96.67%, 94.05%, 89.64%, 96.43%, and 90.71%. However, the results are different for the case of subject **AY**. For **AY**, the highest classification accuracy of 98.69% is attained RSM with RF and 98.45% is attained by the RSM with C4.5. The RoF with C4.5 is the third with an accuracy of 97.14%. RSM with RT is the fourth one with an accuracy of 97.02%. RSM with k-NN is the eighth with an accuracy of 92.38%.

While considering the case of each subject, the highest accuracy of 98.69% is achieved by the RSM with RF. However, for all five subjects, the highest classification accuracy of 94.83% is achieved by the RoF with k-NN. It shows that, in general, the used assembly of MSPCA, WPD, and statistical feature selection using RoF with k-NN results in the best classification performance for the studied dataset.

## 5. Discussion

The results, outlined in the above section, show that, for most of the cases, the proposed framework of MSPCA, WPD, statistical features selection, and RoF with k-NN leads towards a high classification accuracy. However, the best results obtained for the subject **AY** are obtained for a combination of MSPCA, WPD, and statistical feature selection using RSM with RF. It happens due to the variation in EEG signals magnitudes and response time of subjects while executing an MI task. It has an impact on the shape of EEG signals as well as the performance of the postsegmentation, denoising, feature extraction, and classification algorithms. Therefore, various subjects have varying classification accuracy as a result of this.

The BCI is a well-explored domain, and making a performance comparison with state of the art is a tedious task. It is mainly because of the variety of datasets, preprocessing, features extraction, dimension reduction, and classification techniques used in the previous studies. However, a performance comparison of the suggested framework is made with state-of-the-art solutions using similar datasets.  Table 2 provides a review of those studies. It indicates that the suggested method ensures a comparable or superior performance as compared to the previously presented methods. It indicates that the devised denoising, dimension reduction, and ensemble classification approaches have a substantial influence on the overall precision and performance of the system. The self-configurability of ensemble classifiers, as a function of the utilized training dataset, is one of their main advantages. The use of event-driven tools can help in enhancing the computational effectiveness of the suggested method [45–48]. In the future, this aspect can be investigated. The developed system has the potential to be integrated into the future generation of Brain-Computer Interface systems. The solution performed well for the intended dataset. Future work is to test its applicability for other potential Motor Imagery datasets. The incorporation of deep learning tools is another axis to explore.

## 6. Conclusion

In this paper, a novel automated Motor Imagery tasks classification method is proposed. The EEG signals are processed to distinguish between two categories of the brain activities. This approach is an intelligent combination of ensemble learning, Wavelet Packet Decomposition, Multiscale Principal Component Analysis, and subbands statistical features extraction. Results have shown its effectiveness in classifying the intended Motor Imagery tasks. Using an intelligent ensemble of the Random Subspace classifier with Random Forest, the highest subject-dependent accuracy of 98.69% is realized. The suggested ensemble of the Rotation Forest classifier with k-NN achieved the highest subject-independent accuracy of 94.83%.

## Figures and Tables

**Figure 1:** The system block diagram.

**Figure 2:** The employed WPD scheme.

**Figure 3:** The general framework of ensemble classifiers.

**Figure 4:** (a) The EEG signal and (b) denoised version of EEG signal.

**Figure 5:** The 16 subbands, obtained with WPD.

**Figure 6:** Accuracy of different classifiers.

**Figure 7:** F-measure of different classifiers.

**Figure 8:** AUC of different classifiers.

**Table 1:** Summary of the classification performance measures.

Subj.	Classifier	Accuracy		F-measure		AUC	
AA		RSM	RoF	RSM	RoF	RSM	RoF
	SVM	89.64	90.60	0.896	0.906	0.958	0.929
	k-NN	93.45	96.67	0.935	0.967	0.988	0.985
	RF	82.02	84.76	0.820	0.848	0.900	0.928
	C4.5	67.50	74.76	0.675	0.748	0.764	0.834
	REP tree	69.88	67.50	0.699	0.675	0.765	0.746
	RT	70.83	74.29	0.706	0.742	0.799	0.827

**AL**	SVM	86.43	84.88	0.864	0.849	0.923	0.879
	k-NN	92.26	94.05	0.923	0.940	0.970	0.968
	RF	75.00	77.26	0.750	0.773	0.830	0.852
	C4.5	71.07	73.69	0.711	0.737	0.786	0.812
	REP tree	68.93	68.69	0.689	0.687	0.751	0.756
	RT	70.95	70.60	0.708	0.703	0.778	0.786

**AV**	SVM	87.02	84.40	0.870	0.844	0.928	0.886
	k-NN	88.93	89.64	0.889	0.896	0.955	0.939
	RF	73.69	76.90	0.737	0.769	0.818	0.857
	C4.5	61.90	71.31	0.619	0.713	0.677	0.767
	REP tree	62.38	66.19	0.624	0.662	0.671	0.721
	RT	65.00	65.95	0.644	0.654	0.691	0.738

**AW**	SVM	86.90	85.00	0.869	0.850	0.926	0.876
	k-NN	94.64	96.43	0.946	0.964	0.983	0.976
	RF	77.02	78.81	0.770	0.788	0.844	0.867
	C4.5	67.62	71.19	0.676	0.712	0.727	0.788
	REP tree	63.45	68.33	0.634	0.683	0.683	0.742
	RT	68.69	70.24	0.685	0.700	0.735	0.780

**AY**	SVM	92.02	91.90	0.920	0.919	0.984	0.942
	k-NN	92.38	90.71	0.924	0.907	0.977	0.952
	RF	98.69	94.29	0.987	0.943	0.999	0.991
	C4.5	98.45	97.14	0.985	0.971	0.999	0.995
	REP tree	95.60	93.10	0.956	0.931	0.988	0.980
	RT	97.02	93.10	0.970	0.931	0.996	0.985

**ALL**	SVM	89.98	90.12	0.900	0.901	0.962	0.932
	k-NN	93.55	94.83	0.935	0.948	0.984	0.974
	RF	80.36	81.83	0.804	0.818	0.889	0.901
	C4.5	68.57	73.00	0.686	0.730	0.769	0.815
	REP tree	68.60	69.02	0.686	0.690	0.765	0.760
	RT	72.57	72.40	0.724	0.722	0.807	0.809

**Table 2:** Comparison with previous studies.

Study	Feature extraction	Classifier	Classes/subject(s)	Accuracy (%)
[18]	Rényi min-entropy	RF	4/subject independent	80.55
[21]	Subbands PSDs	DNN	2/subject independent	82.48
[37]	Tangent space mapping	SVM	2/1-subject	97.80
[38]	Common spatial pattern	Backpropagation Neural network	2/subject independent	80.73
[39]	Regularized common spatial pattern	SVM	2/subject independent	91.9
[40]	Fisher ratio of time domain parameters	SVM	2/subject independent	89.13
[41]	Common spatial pattern	SVM	2/subject independent	85.01
[42]	Stacked autoencoders (SAE)	CNN	2/subject independent	82.00
[43]	Inverse problem through beamforming	CNN	2/subject independent	90.50
[44]	Granger causality channel selection and common spatial pattern	Linear SVM	2/subject independent	88.46
Proposed	WPD	RF and RSM	2/subject dependent	98.69
	WPD	k-NN and RoF	2/subject independent	94.83

## Data Availability

The dataset used in this paper is publicly available via the following link: http://www.bbci.de/competition/iii/desc_IVa.html.
